# Effect of Pixel’s Spatial Characteristics on Recognition of Isolated Pixelized Chinese Character

**DOI:** 10.2174/1874120701509010234

**Published:** 2015-08-31

**Authors:** Kun Yang, Shuang Liu, Hong Wang, Wei Liu, Yaowei Wu

**Affiliations:** 1 College of Quality and Technical Supervision, Hebei University, 180 Wusidong Road, Baoding, Hebei Province, Chi-na; 2 College of Electronic Information Engineering Hebei University180 Wusidong Road, Baoding, Hebei Province, China

**Keywords:** Pixelized Chinese character, recognition, simulated prosthestic vision, spatial characteristics

## Abstract

The influence of pixel’s spatial characteristics on recognition of isolated Chinese character was investigated using simulated prosthestic vision. The accuracy of Chinese character recognition with 4 kinds of pixel number (6*6, 8*8, 10*10, and 12*12 pixel array) and 3 kinds of pixel shape (Square, Dot and Gaussian) and different pixel spacing were tested through head-mounted display (HMD). A captured image of Chinese characters in font style of Hei were pixelized with Square, Dot and Gaussian pixel. Results showed that pixel number was the most important factor which could affect the recognition of isolated pixelized Chinese Chartars and the accuracy of recognition increased with the addition of pixel number. 10*10 pixel array could provide enough information for people to recognize an isolated Chinese character. At low resolution (6*6 and 8*8 pixel array), there were little difference of recognition accuracy between different pixel shape and different pixel spacing. While as for high resolution (10*10 and 12*12 pixel array), the fluctuation of pixel shape and pixel spacing could not affect the performance of recognition of isolated pixelized Chinese Character.

## 1. INTRODUCTION

Advance in computer technology, biomedical engineering and microelectronics have facilitated the development of supporting or replacing the function of defective tissues or organs with electrical devices. Currently, several visual prostheses approaches have been proposed and have made rapid progress [1-2]. Through stimulation between microelectrode and neural elements, most of visual prostheses have been successful in providing phosphenes perception to subjects. During electrical stimulation studies of the occipital cortex, retina and optic nerve, some blind subjects have been allowed to recognize shapes and letters by phosphenes with correct spatial patterns [13, 14].

However, the models of visual prostheses which could be implemented remain very crude and even more imprecise. Besides the biocompatibility, long-term effectiveness and safety threshold values of implanted electrodes need to be considered cautiously. Low resolution owing to the restricted number of phosphenes severely restricts the performance of visual prostheses. Patient percepts of a letter H and a small box could be created by a stimulation of the retinal surface with an array of 25 electrodes [14], but the stimulation would not allow a blind person to perceive detailed images. Researchers were interested in how to fully explore the utility from a visual prostheses and finding the most valuable data with a limited number of pixels.

Reading is among the most important visual tasks in daily life and also is a main cognitive ability for the blind wearing visual prostheses. Several research groups have been investigating reading with limited number of pixels [15-20]. These previous studies investigated the influence of several parameters of pixels on pixelized reading including: pixel number, pixel size, pixel pitch, grid size and gray level, *et al.* All of these researches focused on pixelized reading of Latin words, while Chinese character doesn't get enough attention. It is well-known that 30% of people all over the world speak Chinese. There are almost 8.77 million Chinese having visual disabilities and each year 450,000 patients become totally blind [21]. It is very important to investigate the performance of visual prostheses on pixelized reading of Chinese character.

Spatial characteristics of the pixel could affect the performance of object recognition using simulated visual prostheses [22-25]. Robert W. Thompson, *et al. *[22] found that grid size, dot size, gap width, dot dropout rate, and gray-scale resolution influenced the discrimination speed and performance of face recognition. Jasmine S. Hayes, *et al. *[23] studied the recognition of object with square and Gaussian pixels array. As for pixelized Latin words reading, Ange´lica and his colleagues [24] discovered that a restricted range of Gaussian widths for which performances were equivalent or significantly better than that obtained with square pixelization. Chinese character is a kind of pictograph which is quite different to English alphabet. Further studies are still necessary for the influence of pixel spatial characteristics on recognition of Chinese characters.

The intention of the research is to study the effect of pixel’s spatial characteristics on recognition of pixelized isolated Chinese character using simulated prosthetics vision in sighted individuals: the influences of (1) pixel number, (2) pixel shape and (3) pixel spacing on the recognition of isolated Chinese character. We test the accuracy of Chinese character recognition with 4 kinds of pixel array number (6*6, 8*8, 10*10, and 12*12 pixel array), 3 kinds of pixel shapes (Square, Dot and Gaussian) and different pixel spacing (four models).

## 2. MATERIALS AND METHODS

### 2.1 Experimental Set-up

The experimental Set-up consist of a head-mounted display (HMD) (iTheater VisionTech Ltd, 2 TFT LCD displays, 320*240 resolution, QVGA, 25° viewing angle, 2.5M at 55’’ screen image size) and a Dell personal computer (2.4GHz CPU, 512MHz DDR RAM) with a self-developed experimental program written in C++ language. Irrelevant visual interference can be reduced by the HMD, such as ambient light and instability of visual angle. Visual angel less than 10° is appropriate for Chinese character recognition [14]. In order to get optimized recognized result, we make 10° as visual angle for every inactive isolated character. The pixelized image of Chinese Character with different pixel parameters was rendered on head-mounted display screen one after another. In the same way, reference information (*e.g. *the pixel number, high resolution character image) rendered on computer screen in very small size. For subjects, they won’t be able to identify the reference information rendered on HMD screen because of the small visual angle, at the same time. The full information of the experimental characters comes to the test administrator.

Pixelized image of Chinese character rendered on the screen of head-mounted display (HMD) and computer simultaneously. The reference information about pixel number, pixel shape, pixel spacing model and a high resolution imaging of character were rendered on the screen of computer in very small size. The subjects were asked to say the character if it is legible, if not, say “no” to the administrator. The recognized results were recorded by the administrator according to subject’s judgment by pressing the key “left” or “right”.

### 2.2 Subjects

Forty volunteers aged between 21 and 36 years from the staff of the Shanghai Jiao Tong University were recruited as volunteers. All volunteers with normal or corrected-to-normal vision and were native Chinese. Each tested subject had fully understood the purpose and procedures before the formal experiment. A launched training program aimed at making the subjects familiar with the experiment.

### 2.3 Processing of Chinese Character

In this experiment, all Chinese characters come from two government-sponsored character lists: (1) The first set of GB 2312-80 International Standard Code which contains 3755 Chinese characters is promulgated by Standardization Administration of China and (2) the List of Frequently Used Characters in Modern Chinese jointly recommended by the National Working Committee on Languages and Writing Systems and the Ministry of Education, China in 1988 which includes 3,500 characters. In order to minimize the familiarity effect, the selection of experimental characters was narrowed in the 631 most commonly used characters, which expresses 80% information of Chinese daily reading. 

With uniformed stroke width, straight horizontal and vertical stroke, Hei font which is one of the most commonly used print font in Chinese made itself the best choice as the experimental character in this experiment to minimize any unexpected confounding effects. Chinese characters were pixelized according to the following procedures: (A) “Microsoft Word” and “ACDSee” were adopted to obtain the original isolated Chinese character bitmap image with a matrix form of 128*128. All Characters were black with white background. (B) In order to get binary images of Chinese characters, a threshold of 150/255 was set. The bitmap image was scanned progressively to get the color of pixels, the pixel value would be set as “1” if the value of gray-scale is higher than the threshold, otherwise it would be set as “0”. (C) The binary image was divided into square zones in same size. The number of zones is consistent with the preset pixel number, for example, a matrix form of 6*6, 8*8, 10*10, and 12*12. If the number of pixel value “1” in each zone was more than 50% of the total pixel number in the zone, “1” would be assigned to represent the whole zone, otherwise “0” would be assigned instead. In order to simulate the real light stimulation, pixels with values of “1” and “0” were rendered as white and black respectively against a black background on the visual screen of HMD. Square pixelized image was acquired with processing above-mentioned. Dot pixelization and Gaussian pixelization was performed by replacing the square zones with Dot pixels and Gaussian pixels (Fig. **1**). 

### 2.4 Experiment 1

The purpose of experiment 1 is to study the effect of pixels number and pixels shape on recognition of isolated pixelized Chinese character. 120 characters were selected from the most frequently used 631 Chinese character. All characters were pixelized into 6*6, 8*8, 10*10 and 12*12 pixels array with three shape models (Square, Dot and Gaussian), experimental sample seen Fig. (**2**).

To avoid memory and learning effect, the subjects were tested from low to high resolution. The testing order of the pixel arrays was 6*6, 8*8, 10*10, and 12*12. A training program was launched in order to make the subjects familiar with the experimental process. Pixelized characters were rendered on both screens of computer and HMD in sequence against black background. Each subject was requested to pronounce the character if it was legible, if not, tell the administrator “no”. The administrator recorded the results according to participant’s judgment by pressing the key “left” or “right”, where “left” means correct and “right” means illegibility or wrong. The experimental program records the results and calculates recognition accuracy.

### 2.5 Experiment 2

The purpose of experiment 2 is to study the effect of pixels spacing on recognition of isolated pixelized Chinese character. 120 characters were selected from the 631 most commonly used Chinese character and pixelized into 6*6, 8*8, 10*10 and 12*12 pixels array with Dot pixel. The pixel spacing was set into four models (Fig. **3**): Model 1: the spacing between neighboring pixels was zero; Model 2: the diameter of pixel was 3/4 of model 1, and the spacing between neighboring pixels was 33% of pixel diameter; Model 3: the diameter of pixel was 1/2 of model 1, and the spacing between neighboring pixels was 100% of pixel diameter; Model 4: the diameter of pixel was 1/4 of model 1, and the spacing between neighboring pixels was 300% of pixel diameter. The experimental procedure was similar to experiment 1.

## 3. RESULTS AND DISCUSSION

As shown in Fig. (**4**), the pixel number has effected remarkably on recognition accuracy of Chinese characters. The recognition accuracy increased with the resolution for all the three pixel shapes. Table **1** lists the values of recognition accuracy according to different pixel number and pixel shapes.

Higher recognition accuracy was achieved with Gaussian pixels than the other two models at 6*6 and 8*8 pixel array. That means Chinese characters with Gaussian pixels were much more legible than that with Dot pixels and Square pixels. The difference of accuracy between these models was significant for low resolution (6*6, 8*8 pixel array), while insignificant for high resolution (10*10, 12*12 pixel array). 

Fig. (**5**) reveal the accuracy of Chinese character recognition with four pixel models in 6*6, 8*8, 10*10 and 12*12 pixel array. There was no remarkable difference between the four models at high resolution (10*10 and 12*12 pixels array); more than 90% Chinese characters could be recognized correctly for all four models. At low resolution (6*6 and 8*8 pixel array), the accuracy of model 1 was a little smaller than that of the other three models. Table **2** lists the values of recognition accuracy according to different models.

Some unavoidable factors, such as physical and mental state, personal knowledge and experience, may have the influence on the results in the study. A detailed introduction and pre-training were conducted before the test in order to eliminate the subjects’ worries. We offered two short breaks during the period of test to make the subjects relaxed and reduce the fatigue caused by long time experiment. Although the effects of psychological factors cannot be removed completely, we have tried to reduce them to the minimum. 

The HMD and totally black background eliminate the effects of luminance distributions and background noise. The most frequently Used Chinese characters were chosen, so that each character could be easily recognized as soon as it was legible. The influence of knowledge background and educational level of the subjects can also be minimized in our experimental results. The testing order of pixelized Chinese character was designed from low resolution (6*6 pixel array) to high resolution (12*12 pixel array) in order to minimize learning and memory effects on the results.

We reduced the number of descriptors and focus our experiment on the impact of pixel’s spatial Characteristic (pixel number, pixel shape, pixel spacing). The result of Experient1 indicates that the pixel number was the most important factor on recognition of pixelized Chinese Characters. Pixel shape may be a critical issue for the prosthetic vision. Phosphenes elicited by electrical stimulation of the retina should not be of constant luminosity and not of square shape. The results of Experiment 1 indicated that the pixel shape affects the recognition accuracy only at low resolution (6*6 pixel array). As for high resolution (no less than 10*10 pixel array), there are almost no difference between the three shapes. Since the 10*10 pixel array was the minimum requirement for recognition of pixelized Chinese Character, the results mean any one of pixel shapes (Square, Dot and Gaussian) was suitable for this purpose.

The strength of stimulation current effects the patterns of neural activity which elicited by electric stimulation and that neural activation diminishes progressively with increasing of electrode-to-neural target distance [26-29]. There are possible spacing or overlap between neighboring phosphenes according to the strength of the stimulation current. The results of Experiment 2 were very interesting and also different to our anticipation. It was expected that the recognition accuracy drops down with the increase of pixel spacing. While the results show that the recognition accuracy of model 1 was less than that of the other three models at low resolution (6*6 and 8*8 pixel array). Whereas at high resolution (10*10 and 12*12 pixel array), the recognition accuracy was of no difference between the four spacing models. Possible reasons are that the Chinese character was a kind of pictograph, and that the stroke and the structure are the most important factors for the identification. Low resolution provide limited information for recognition of Chinese character, furthermore the big pixel size affect the identification of structures especially for some radical combination structures, such as left–right (*e.g.*,), up–down (*e.g.*,), P-shaped (*e.g.*,), L-shaped (*e.g.*,), and enclosed (*e.g.*,) structures. At high resolution, the pixel size decreased with the increase of pixel spacing which results in illegibility of Chinese character. Nevertheless, higher resolution provides sufficient information so that the stroke and the structure could be identified. 

For future visual prostheses based on point-to-point interconnection between micro-electrode contacts and neural elements, the pixel size and the spacing of neighboring pixels depend on the strength of stimulation current. High stimulation current results in big pixel size and small spacing or overlap, while low stimulation current results in small pixel size and big spacing. The experiment presented a simulated test in sighted individuals so that there should be some difference between the vision produced by the visual prostheses and simulated prosthestic vision. Despite these limitations, we hope this study could provide useful reference for development of visual prostheses.

## CONCLUSION

In this study, the influences of spatial characteristic on recognition of Chinese character were investigated. The results indicated that pixel number, pixel shape and pixel spacing all have influence on legibility of isolated pixelized Chinese character. Pixel number plays the most important role in recognition of pixelized Chinese character using simulated prosthestic vision. The recognition accuracy of pixelized Chinese character increased greatly with pixel number. The minimum requirement for recognition of isolated Chinese character is 10*10 pixel array. The three pixel shapes (Square, Dot and Gaussian) provide almost same performance at high resolution (10*10, 12*12 pixel array). The Gaussian shape obtained higher recognition accuracy at low resolution (6*6 and 8*8 pixel array). There is no remarkably difference of recognition of pixelized Chinese Character between different spacing models of neighboring pixels at 10*10 and 12*12 pixel array. The recognition accuracy of model 1 (zero pixel spacing) was the least among the four models at 6*6 pixel array. 

## Figures and Tables

**Fig. (1):** Experimental sample of pixelized character: (A) Original image of Chinese character, (B) Reversed color image, (C) Character with 12*12 Square pixel array, (D) Character with 12*12 Dot pixel array, (E) Character with 12*12 Gaussion pixel array.

**Fig. (2):** Sample images used in this experiment. Each column corresponds to a given number of pixels (6*6, 8*8, 10*10, and 12 *12) and each row corresponds to a pixel shape. Visual angle of each character image was set in 10°.

**Fig. (3):** Sample images used in this experiment. Each column corresponds to a given number of pixels (6*6, 8*8, 10*10, and 12*12) and each row corresponds to a pixel spacing model.

**Fig. (4):** The accuracy of Chinese character recognition with 4 kinds of pixel array number (6*6, 8*8, 10*10, and 12*12) and 3 kinds of different pixel shape (Square, Dot and Gaussian).

**Fig. (5):** Accuracy of Chinese character recognition with different pixels spacing model. (A) 6*6 pixel array, (B) 8*8 pixel array, (C) 10*10 pixel array, (D) 12*12 pixel array.

**Table 1.** Mean accuracy of Chinese character recognition with different pixel number and pixel shape.

	6*6	8*8	10*10	12*12
Gaussian	39.78±5.19%	73.70±8.85%	92.90±5.69%	98.55±1.98%
Dot	31.67±7.02%	69.71±10.37%	90.58±7.82%	98.33±2.14%
Square	28.40±4.05%	69.75±7.23%	91.98±3.86%	98.29±1.41%

**Table 2.** Mean accuracy of Chinese character recognition with different pixel.

	6*6	8*8	10*10	12*12
Model 1	31.67±7.02%	69.71±10.37%	90.58±7.82%	98.33±2.14%
Model 3	40.14±6.83%	70.94±9.86%	90.87±6.83%	97.32±2.54%
Model 3	39.64±5.79%	72.83±9.12%	92.39±6.29%	98.55±2.47%
Model 4	38.70±5.29%	72.10±9.48%	91.74±6.36%	98.70±1.39%

## References

[1] Brelén M.E., Duret F., Gérard B., Delbeke J., Veraart C. (2005). Creating a meaningful visual perception in blind volunteers by optic nerve stimulation.. J. Neural Eng..

[2] Chow A.Y., Chow V.Y. (1997). Subretinal electrical stimulation of the rabbit retina.. Neurosci. Lett..

[3] Delbeke J., Oozeer M., Veraart C. (2003). Position, size and luminosity of phosphenes generated by direct optic nerve stimulation.. Vision Res..

[4] Dobelle W.H. (2000). Artificial vision for the blind by connecting a television camera to the visual cortex.. ASAIO J..

[5] Humayun M.S., de Juan E. (1998). Artificial vision.. Eye (Lond.).

[6] Humayun M.S., Weiland J.D., Fujii G.Y., Greenberg R., Williamson R., Little J., Mech B., Cimmarusti V., Van Boemel G., Dagnelie G., de Juan E. (2003). Visual perception in a blind subject with a chronic microelectronic retinal prosthesis.. Vision Res..

[7] Normann R.A., Maynard E.M., Rousche P.J., Warren D.J. (1999). A neural interface for a cortical vision prosthesis.. Vision Res..

[8] Rizzo J.F., Wyatt J., Loewenstein J., Kelly S., Shire D. (2003). Perceptual efficacy of electrical stimulation of human retina with a microelectrode array during short-term surgical trials.. Invest. Ophthalmol. Vis. Sci..

[9] Rizzo J.F., Wyatt J. (1997). Prospects for a visual prostheses.. Neuroscientist.

[10] Veraart C., Raftopoulos C., Mortimer J.T., Delbeke J., Pins D., Michaux G., Vanlierde A., Parrini S., Wanet-Defalque M.C. (1998). Visual sensations produced by optic nerve stimulation using an implanted self-sizing spiral cuff electrode.. Brain Res..

[11] Zrenner E. (2002). Will retinal implants restore vision?. Science.

[12] Zrenner E., Stett A., Weiss S., Aramant R.B., Guenther E., Kohler K., Miliczek K.D., Seiler M.J., Haemmerle H. (1999). Can subretinal microphotodiodes successfully replace degenerated photoreceptors?. Vision Res..

[13] Dobelle W.H., Mladejovsky M.G., Evans J.R., Roberts T.S., Girvin J.P. (1976). “Braille” reading by a blind volunteer by visual cortex stimulation.. Nature.

[14] Humayun M.S., de Juan E., Weiland J.D., Dagnelie G., Katona S., Greenberg R., Suzuki S. (1999). Pattern electrical stimulation of the human retina.. Vision Res..

[15] Legge G.E., Pelli D.G., Rubin G.S., Schleske M.M. (1985). Psychophysics of reading--I. Normal vision.. Vision Res..

[16] Cha K., Horch K.W., Normann R.A., Boman D.K. (1992). Reading speed with a pixelized vision system.. J. Opt. Soc. Am. A.

[17] Dagnelie G., Thompson R.W., Barnett G.D., Zhang W.Q. (2000). Visual perception and performance under conditions simulating prosthetic vision.. Perception.

[18] Sommerhalder J., Oueghlani E., Bagnoud M., Leonards U., Safran A.B., Pelizzone M. (2003). Simulation of artificial vision: I. Eccentric reading of isolated words, and perceptual learning.. Vision Res..

[19] Sommerhalder J., Rappaz B., de Haller R., Fornos A.P., Safran A.B., Pelizzone M. (2004). Simulation of artificial vision: II. Eccentric reading of full-page text and the learning of this task.. Vision Res..

[20] Fu L., Cai S., Zhang H. (2006). Psychophysics of reading with a limited number of pixels: Towards the rehabilitation of reading ability with visual prostheses.

[21] Chai X., Yu W., Wang J., Zhao Y., Cai C., Ren Q. (2007). Recognition of pixelized Chinese characters using simulated prosthetic vision.. Artif. Organs.

[22] Thompson R.W., Barnett G.D., Humayun M.S., Dagnelie G. (2003). Facial recognition using simulated prosthetic pixelized vision.. Invest. Ophthalmol. Vis. Sci..

[23] Hayes J.S., Yin V.T., Piyathaisere D., Weiland J.D., Humayun M.S., Dagnelie G. (2003). Visually guided performance of simple tasks using simulated prosthetic vision.. Artif. Organs.

[24] Weiland J.D., Humayun M.S., Dagnelie G., de Juan E., Greenberg R.J., Iliff N.T. (1999). Understanding the origin of visual percepts elicited by electrical stimulation of the human retina.. Graefes Arch. Clin. Exp. Ophthalmol..

[25] Stett A., Barth W., Weiss S., Haemmerle H., Zrenner E. (2000). Electrical multisite stimulation of the isolated chicken retina.. Vision Res..

[26] Rizzo J.F., Wyatt J., Loewenstein J., Kelly S., Shire D. (2003). Perceptual efficacy of electrical stimulation of human retina with a microelectrode array during short-term surgical trials.. Invest. Ophthalmol. Vis. Sci..

[27] Fornos A.P., Sommerhalder J., Rappaz B., Safran A.B., Pelizzone M. (2005). Simulation of artificial vision, III: do the spatial or temporal characteristics of stimulus pixelization really matter?. Invest. Ophthalmol. Vis. Sci..

[28] Yang K., Zhou C., Ren Q., Fan J., Zhang L., Chai X. (2010). Complexity analysis based on image-processing method and pixelized recognition of Chinese characters using simulated prosthetic vision.. Artif. Organs.

[29] Zhou Y., Lu Y., Tian Y., Li L., Ren Q., Chai X. (2010). Image processing based recognition of images with a limited number of pixels using simulated prosthetic vision.. Inf. Sci..

